RETRACTED

# METTL3 enhances the effect of YTHDF1 on *NEDD1* mRNA stability by m6A modification in diffuse large B‐cell lymphoma cells

**DOI:** 10.1002/iid3.789

**Published:** 2023-02-24

**Authors:** Lili Feng, Qinying Yan, Hui Pan, Wodong Shi

**Affiliations:** ^1^ Department of Ophthalmology, Shanghai Ninth People's Hospital Shanghai Jiao Tong University School of Medicine Shanghai China; ^2^ College of Pharmaceutical Sciences Zhejiang University of Technology Hangzhou China

**Keywords:** diffuse large B‐cell lymphoma, METTL3, NEDD1, the Hedgehog signaling, YTHDF1

## Abstract

**Aim:**

Diffuse large B‐cell lymphoma (DLBCL) remains the most frequent subpopulation of lymphoma, and N6‐methyladenosine (m6A) was implicated in the DLBCL progression. Herein, we sought to decipher the m6A‐asociated mechanism of *NEDD1* in DLBCL development.

**Methods:**

The NEDD1 expression profile in DLBCL was assessed by quantitative real‐time polymerase chain reaction (RT‐qPCR) and Western blot. NEDD1 was artificially downregulated or upregulated in DLBCL cells, followed by EdU, Transwell assays and flow cytometry. The Hedgehog pathway activity was assayed by a dual‐luciferase assay. The m6A methylation of *NEDD1* in DLBCL was assessed by meRIP‐qPCR, and the regulatory mechanism of METTL3 on *NEDD1* was validated. The LDH assay was conducted to examine the impact of CD8^+^ T cells on DLBCL cells. The DLBCL cells were administrated into mice to evaluate the tumorigenic activity and ki‐67 activity in tumor tissues.

**Results:**

NEDD1 was overexpressed in DLBCL. Depletion of *NEDD1* inhibited the aggressiveness of SU‐DHL‐8 and OCI‐LY1 cells, whereas overexpression of *NEDD1* expedited the aggressiveness of SU‐DHL‐8 and OCI‐LY1 cells. METTL3 promoted *NEDD1* translation in an m6A‐dependent manner via YTHDF1. Depletion of *METTL3* inhibited SU‐DHL‐8 and OCI‐LY1 cell activity through regulation of *NEDD1*. *NEDD1* reversed the repressive effect of *METTL3* loss on the aggressiveness of SU‐DHL‐8 and OCI‐LY1 cells. *NEDD1* activated the Hedgehog signaling to promote immune escape of DLBCL.

**Conclusions:**

METTL3 promotes translation of *NEDD1* via YTHDF1‐depedndent m6A modification, thereby activating the Hedgehog signaling pathway to promote immune escape of DLBCL cells.

## Graphical abstract

Our study collectively uncovered that NEDD1 promoted proliferation, invasion, and tumor growth of diffuse large B‐cell lymphoma (DLBCL) in vitro and in vivo.

## 1 INTRODUCTION

Large B‐cell lymphomas, with a projected 150,000 new diagnoses annually worldwide, represent near 30% of non‐Hodgkin's lymphoma cases.^1^ Most patients with diffuse large B‐cell lymphoma (DLBCL) can be cured with standard rituximab, cyclophosphamide, doxorubicin, vincristine, and prednisone, while patients who fail this front‐line therapy have a dismal outcome.^2^ Targeting cancer cells via the modulation of the immune system has become a new therapeutic option in many different malignancies, including lymphoma.^3^, ^4^, ^5^ Among them, chimeric antigen receptor T cells, bispecific T cell engagers, immunomodulatory drugs, and epigenetic‑modifying drugs might offer new opportunities for those relapsed/refractory patients.^6^ The presence of CD8^+^ T cells has been associated with the immune inhibitory mechanism‐mediated immune suppression.^7^ Therefore, further research on CD8^+^ T cell function is necessary for generating new therapeutic strategies in DLBCL.

RETRACTED

Neural precursor cell expressed developmentally downregulated protein 1 (NEDD1) localizes to the centrosome and mitotic spindle, and the localization of key centrosomal proteins is imperative in preventing cells against uncontrolled growth and the development of cancers, suggesting that NEDD1 might be a possible candidate for anticancer treatment.^8^ Moreover, NEDD9 overexpression was related to genetic abnormalities and prognosis and might serve as a possible biomarker guiding the choice between hematopoietic stem cell transplantation and chemotherapy in patients with acute myeloid leukemia after achieving complete remission.^9^ However, there is little evidence showing the direct linkage between NEDD1 overexpression and the development of DLBCL. Critically, the N6‐methyladenosine (m6A)‐based prognostic signature has been reported to be a prognostic predictor for DLBCL, and immune microenvironment governed by m6A might be a part of the mechanism.^10^ The significance of m6A, the most abundant mRNA modification, has emerged in the field of biology science for the discovery of its “writers,” “erasers,” and “readers” that can add, remove, or bind to the m6A site, thus manipulating imperative biological function.^11^, ^12^, ^13^ For instance, methyltransferase 3 (METTL3), a well‐known writer, modulated the expression of *Epstein‐Barr nuclear antigen 2* during Epstein–Barr virus infection.^14^ Under the context of DLBCL, METTL3 deletion abated the m6A methylation modification and mRNA expression of *pigment epithelium‐derived factor*.^15^ The importance of the sonic hedgehog signaling to DLBCL has been described in a previous study.^16^ On the basis of these findings, we postulated here that the NEDD1 expression in DLBCL was also regulated by the METTL3‐mediated m6A modification. This research aimed at probing the regulation of METTL3 on NEDD1 expression and DLBCL cell immune escape via Hedgehog signaling.

RETRACTED

## 2 MATERIALS AND METHODS

### 2.1 Tissues

Lymph node tissues were obtained from 24 patients with DLBCL diagnosed at Shanghai Ninth People's Hospital from January 2018 to August 2019. Tumor‐infiltrating tissues and nonneoplastic tissues were separated in an ultra‐clean bench. All samples were histologically examined before the experiment and confirmed to be tumor‐infiltrating tissues and nonneoplastic tissues, respectively. There were 15 male patients and nine female patients, aged 40–80 years, with a median age of 58 years. Seven patients were of the germinal center B‐cell‐like (GCB) type and 17 patients were of the non‐GCB type. A proportion of specimens was rapidly placed in a −80°C refrigerator for subsequent testing. All these patients had not received radiotherapy or chemotherapy before the tissue collection. This study was approved by the Institutional Review Board of Shanghai Ninth People's Hospital (approval number: 2017‐379‐T277). All patients enrolled in the study signed informed consent.

### 2.2 Cell culture

DLBCL cells SU‐DHL‐8 and OCI‐LY1 were purchased from the ATCC and Shanghai Jingkang Bioengineering Co., Ltd., respectively. A human lymphoblastoid cell line AHH‐1 was acquired from Mingzhoubio. CD8^+^ T cells were purchased from BlueFBio.

SU‐DHL‐8, OCI‐LY1, and AHH‐1 cells were cultured in RPMI‐1640 medium plus 10% fetal bovine serum (FBS), 2 mmol/L l‐glutamine and 100 U/mL penicillin/streptomycin at 37°C in a 5% CO_2_ incubator. CD8^+^ T cells were grown in Dulbecco's modified Eagle's medium plus 10% FBS and 100 units/mL penicillin/streptomycin at 37°C in a 5% CO_2_ incubator. All reagents for cell culture were acquired from Thermo Fisher Scientific Inc.

### 2.3 Cell infection

Lentiviral harboring small interfering RNA (siRNA) plasmids targeting NEDD1 (si‐NEDD1), METTL3 (si‐METTL3), and YTHDF1 (si‐YTHDF1), NEDD1‐overexpression (NEDD1‐OE), an overexpression fragment targeting NEDD1, and the negative controls (NC) were synthesized by Sangon. Lipofectamine 2000 (Thermo Fisher Scientific) was applied for lentivirus packaging. When the cells had grown to an 80%–90% confluence, the Lipo 2000‐DNA mixture was prepared in a certain ratio (1 µg of transfected plasmid: 2.5 µL of Lipo 2000 transfection reagent). In brief, the Lipo 2000 transfection reagent was mixed with 100 µL OPTI‐MEM (Thermo Fisher Scientific) and allowed to stand for 5 min in one tube. In another tube, the total volume of plasmids was mixed with 100 µL OPTI‐MEM. The samples in the two tubes were mixed, centrifuged, and left for 15 min at room temperature. Finally, the total Lipo 2000‐DNA mixture was supplemented to the HEK293T cell culture medium, and the medium was gently shaken and mixed to continue incubation. After 6–8 h, the medium was refreshed with the complete medium containing serum. Cell supernatant was collected 24 h after lentivirus packaging for lentivirus infection of DLBCL cells. The collected lentivirus solution and DLBCL cells were co‐incubated for 48 h, and then the corresponding antibiotics were added for the screening of stable infected cell lines.

RETRACTED

### 2.4 RT‐qPCR

The TRIzol kit (Thermo Fisher) was used for total RNA extraction. A Nano‐drop 2000 spectrophotometer (Thermo Fisher Scientific) was applied to determine the RNA concentration, and 100 ng of RNA was reverse‐transcribed to cDNA using the iScript cDNA Synthesis Kit (Bio‐Rad Laboratories), followed by RT‐qPCR on a 7900HT system (Applied Biosystems) using the SYBR™ GreenER™ qPCR Supermix (Thermo Fisher Scientific). The mRNA expression was normalized to GAPDH and measured using the 2^−ΔΔCt^ method. PCR primers (synthesized by Sangon) were presented below: METTL3 forward 5′‐TTTCCGGTTAGCCTTCGGG‐3′ and reverse 5′‐ATGGACACAGCATCAGTGGG‐3′; YTHDF1 forward 5′‐CGCCAGCTTCAGGGAGATAAA‐3′ and reverse 5′‐TCCCCAATCTTCAGGCCAAC‐3′; NEDD1 forward 5′‐TTGCCTCGTCTCCACAAGTC‐3′ and reverse 5′‐CCCGGGAAGATCCAATAGCC‐3′; GAPDH forward 5′‐AATGGGCAGCCGTTAGGAAA‐3′ and reverse 5′‐GCGCCCAATACGACCAAATC‐3′.

### 2.5 Me‐RIP assay

Extracted total RNA was chemically fragmented and incubated with m6A antibody according to the standard method using the Me‐RIP Kit (Guangzhou RiboBio Co., Ltd.), and immunoprecipitation was performed. RNA was subsequently extracted by proteinase K (Thermo Fisher) for RT‐qPCR analysis.

### 2.6 Western blot analysis

Cells and tissues were lysed with lysis buffer, followed by protein concentration determination using the bicinchoninic acid (BCA) protein assay kit (Thermo Fisher Scientific). After that, 30 µg protein was separated on 10% sodium dodecyl sulfate‐polyacrylamide gel electrophoresis and transferred to polyvinylidene difluoride membranes (Sigma‐Aldrich Chemical Company). After being sealed with 5% nonfat milk, the membranes were probed with primary antibodies including NEDD1 (1:2000, PHN5820, Abmart Shanghai Co., Ltd.), transforming growth factor‐β (TGF‐β 1:1000, #3709, Cell Signaling Technologies (CST)), interleukin (IL)‐10 (1:1000, #12163, CST), METTL3 (1:1000, ab195352) and GAPDH (1:1000, #2118, CST), followed by 1 h of incubation with secondary horseradish peroxidase (HRP)‐labeled goat anti‐rabbit IgG (1:3000, ab205718, Abcam). Blots were visualized using enhanced chemiluminescent detection.

### 2.7 Enzyme‐linked immunosorbent assay (ELISA)

The levels of TGF‐β and IL‐10 in DLBCL cell culture supernatants and mouse tumor tissues were measured with TGF‐β (ml022522‐2, MLBio, Shanghai, China) and IL‐10 (K4167, BioVision, Inc.) kits. Briefly, the OD values at 450 nm of the samples to be tested, and the standards were assessed. Finally, the standard curve was plotted, and the contents of TGF‐β and IL‐10 were calculated according to the standard curve.

RETRACTED

### 2.8 Cell proliferation assay

The cell proliferation assay was performed using Click‐iT™ EdU Cell Proliferation Imaging Kit (C10340, Thermo Fisher). The cells were plated in 96‐well plates at 7 × 10^3^ cells, treated for 2 h at 37°C with 50 mol/L EdU solution, fixed for 30 min using 4% paraformaldehyde, and treated with Triton X‐100 (Thermo Fisher) for 10 min. The cells were reacted for 30 min with Click‐iT reaction solution in the dark before nuclear staining using Hoechst33342 solution (Beyotime). The cell proliferation rate was assessed using the images taken under a fluorescent microscope (Keyence).

### 2.9 Transwell migration and invasion assays

Transwell chambers (Unique) with 8 µm polycarbonate nucleopore filter membranes were used to perform Transwell assays to detect cell migration and invasion. A total of 2.0 × 10^4^ cells in serum‐free medium were loaded into the apical chamber with or without Matrigel (Unique) attached, and a complete medium containing 10% FBS was loaded onto the basolateral chamber. After a 24‐h incubation at 37°C in a 5% CO_2_ incubator, the cells migrated or invaded through the Matrigel underwent fixation using 4% paraformaldehyde, staining with 0.1% crystal violet (Merck Millipore) and observation in five fields of view using a microscope (Leica Microsystems GmbH).

### 2.10 Cell apoptosis assay

The Annexin V‐FITC/PI Apoptosis Detection Kit (Phygene) was utilized to evaluate cell apoptosis. The cells were washed twice with cold phosphate‐buffered saline. After the resuspension of 5.0 × 10^5^ cells in 1x binding buffer, 5 µL Annexin V‐FITC and 10 µL PI were supplemented to 100 µL cells for a 0.5‐h incubation at room temperature in darkness, and the apoptosis rate was determined by FACScan (Bio‐Rad Laboratories).

### 2.11 Dual‐luciferase reporter assay

GLi‐Luc fluorophore enzyme reporter gene plasmid (Yeasen) was introduced into cells treated with si‐NEDD1 or si‐NEDD1 + smoothened agonist (SAG, 59 nM, Sigma‐Aldrich). The dual‐luciferase reporter assay system was used to determine the Hedgehog signaling pathway activity. According to the protocol of the Dual‐Luciferase Reporter Gene Assay Kit (Yeasen), 1X passive lysis buffer was supplemented to the culture plate and lysed on a micro shaker at room temperature for 15 min to fully lyse the cells. The lysate after sufficient lysis was centrifuged at 1000 rpm for 5 min, and the supernatant was transferred into a fresh EP tube. The firefly luciferase activity was normalized to that of Renilla luciferase.

RETRACTED

### 2.12 RNA stability analysis

To determine the stability of RNA, 5 g/mL actinomycin D (Sigma‐Aldrich) was supplemented to the cells and incubated to the designated time points. Total RNA was extracted at each time point and subjected to RT‐qPCR.

### 2.13 Lactate dehydrogenase (LDH) release assay

CD8^+^ T cells after stimulation with CD3/CD28 magnetic beads were cocultured with SU‐DHL‐8 and OCI‐LY1 cells at 2:1, 3:1, or 5:1 ratio. After 24 h, the LDH cytotoxicity kit (Beyotime) was utilized. The OD490 value was read using an iMark microplate reader (Bio‐Rad). CD8^+^ T cell killing effect (%) = (The experimental group − spontaneous LDH release from the effector cells − spontaneous LDH release from the target cells)/(maximum LDH release from the target cells − spontaneous LDH release from the target cells) × 100%.

### 2.14 Mouse xenograft model

Twenty 3–4‐week‐old male C57BL/6 N mice (weighing 14 ± 2 g, Vital River) were housed at 25°C and 45% humidity with food and water ad libitum. All mouse experiments were performed according to National Institutes of Health guidelines. Experimental protocols were approved by the Animal Ethics Committee of Shanghai Ninth People's Hospital (approval number: 20220223). The SU‐DHL‐8 cells at the logarithmic growth were adjusted to 1 × 10^7^ cells/mL. Mice were subcutaneously injected with the mixture of 100 μL cell suspension and 100 μL Matrigel in the axilla. The tumor growth was observed. After 4 weeks, 1% pentobarbital sodium was injected for euthanasia at 150 mg/kg, and the tumors were dissected, photographed, and weighed.

### 2.15 Immunohistochemical labeling

The tissue sections were subjected to a 2‐h incubation at 60°C, dewaxing, and dehydration. The sections were treated with 3% hydrogen peroxide for 10 min, heated with 0.01 M citrate buffer in a microwave oven for 15 min at 98°C, and then cooled at room temperature for 20 min. The sections were incubated with normal serum for 0.5 h, followed by incubation with ki‐67 antibody (1:200, ab16667, Abcam) overnight at 4°C and with HRP‐labeled goat anti‐rabbit IgG (1:3000, ab205718, Abcam) for 60 min at room temperature. The sections were stained with diaminobenzidine (#ZLI‐9017, ZSGB‐Bio) and observed under a microscope (Leica).

### 2.16 Statistics

All experiments were performed in triplicates, and results are displayed as mean ± SD where applicable. SPSS 22.0 software (IBM Corp.) and GraphPad Prism 8 (GraphPad Software) were used for statistical analysis. Comparisons were carried out by paired *t*‐test, one‐way or two‐way ANOVA (with Tukey's post hoc test). A *p* value < .05 was adopted for significance.

RETRACTED

## 3 RESULTS

### 3.1 High expression of NEDD1 is identified in DLBCL

NEDD1 showed significantly high expression in DLBC by GEPIA database analysis (http://gepia.cancer-pku.cn/detail.php?gene=NEDD1) (Figure 1A). Based on RT‐qPCR, we found elevated mRNA levels of *NEDD1* in DLBCL tissues (*n* = 24) of our cohort relative to the nonneoplastic tissues (Figure 1B). Furthermore, the increased protein expression of NEDD1 in DLBCL tissues was confirmed by western blot (Figure 1C).

**Figure 1:** NEDD1 is overexpressed in DLBCL. (A) Expression of NEDD1 in DLBCL (*n* = 47) and normal tissues (*n* = 337) analyzed in the GEPIA database. (B) The mRNA expression of *NEDD1* in DLBCL and nonneoplastic tissues by RT‐qPCR (*n* = 24). (C) The protein expression of NEDD1 in DLBCL and nonneoplastic tissues by western blot. Mean ± SD (paired *t*‐test). *p < .05 versus nonneoplastic or normal group. DLBCL, diffuse large B‐cell lymphoma; mRNA, messenger RNA; RT‐qPCR, quantitative real‐time polymerase chain reaction; SD, standard deviation.

### 3.2 NEDD1 knockdown suppresses DLBCL cell proliferation and mobility

Subsequently, we downregulated or upregulated NEDD1 expression in SU‐DHL‐8 and OCI‐LY1 cells and tested whether alteration of NEDD1 expression affected the proliferation and aggressiveness of DLBCL cells. First, we infected cells with si‐NEDD1 or NEDD1‐OE and verified the infection efficiency using RT‐qPCR and western blot (Figure 2A). Deletion of NEDD1 inhibited the proliferation of SU‐DHL‐8 and OCI‐LY1 cells (Figure 2B). Transwell assays were performed to count migrated, and invasive cells, and silencing of NEDD1 diminished migration and invasion of DLBCL cells (Figure 2C,D). The apoptosis rate of SU‐DHL‐8 and OCI‐LY1 cells infected with si‐NEDD1 was higher than that of the cells infected with si‐NC (Figure 2E). By contrast, overexpression of NEDD1 potentiated the growth, motility, and apoptosis resistance of SU‐DHL‐8 and OCI‐LY1 cells (Figure 2B–E).

**Figure 2:** NEDD1 loss impairs the proliferation of DLBCL cells. (A) NEDD1 expression in DLBCL cells in response to si‐NEDD1 or NEDD1‐OE using RT‐qPCR and western blot. (B) DLBCL cell proliferation examined using EdU assay. (C) DLBCL cell migration measured using Transwell migration assay. (D) DLBCL cell invasion measured using Transwell invasion assay. (E) DLBCL cell apoptosis measured using flow cytometry. Mean ± SD (two‐way ANOVA). *p < .05 versus si‐NC group, #*p* < .05 versus NC‐OE group. ANOVA, analysis of variance; DLBCL, diffuse large B‐cell lymphoma; EdU, 5‐ethynyl‐2′‐deoxyuridine; RT‐qPCR, quantitative real‐time polymerase chain reaction; SD, standard deviation.

RETRACTED

### 3.3 NEDD1 induces the Hedgehog signaling to expedite DLBCL cell immune escape

The impact of NEDD1 on the Hedgehog signaling was examined by a dual‐luciferase reporter system. It was found that silencing of NEDD1 inhibited the luciferase activity of GLi‐Luc and suppressed the activation of luciferase activity of GLi‐Luc by SAG (Figure 3A). Moreover, it was observed that silencing of NEDD1 decreased the protein expression of TGF‐β and IL‐10 in SU‐DHL‐8 and OCI‐LY1 cells (Figure 3B). It was also revealed by ELISA that silencing of NEDD1 led to a decline in TGF‐β and IL‐10 levels in the cell supernatant (Figure 3C).

**Figure 3:** NEDD1 activates the Hedgehog pathway to promote DLBCL immune escape. (A) The activity of GLi‐Luc in DLBCL cells in response to si‐NEDD1 alone or with SAG using a dual‐luciferase reporter system. (B) The protein expression of immunosuppressive factors TGF‐β and IL‐10 in DLBCL cells in response to si‐NEDD1 using western blot. (C) The levels of TGF‐β and IL‐10 in DLBCL cells in response to si‐NEDD1 using ELISA. (D) The killing effect of CD8^+^ T cells on DLBCL cells in response to si‐NEDD1 using LDH assay. Mean ± SD (two‐way ANOVA). *p < .05 versus si‐NC or coculture + si‐NC group; #*p* < .05 versus si‐NC + SAG group. ANOVA, analysis of variance; DLBCL, diffuse large B‐cell lymphoma; IL, interleukin; LDH, lactate dehydrogenase; SD, standard deviation; TGF‐transforming growth factor.

To further understand whether NEDD1 affects immune escape, we used an LDH cytotoxicity kit. The results showed that depletion of NEDD1 potentiated the killing effect of CD8^+^ T cells on SU‐DHL‐8 and OCI‐LY1 cells, and the promotion was more pronounced with the increase in the proportion of CD8^+^ T cells in the coculture system (Figure 3D).

### 3.4 METTL3 regulates *NEDD1* expression through m6A modification

We analyzed the m6A methylation of *NEDD1* mRNA in DLBCL tissues. The m6A methylation level of *NEDD1* was remarkably increased in DLBCL tissues relative to nonneoplastic tissues (Figure 4A). DLBCL cells displayed higher levels of m6A modification than AHH‐1 cells (Figure 4B), suggesting that *NEDD1* m6A modification might be involved in the pathogenesis of DLBCL. In the GEPIA database, Pearson's correlation analysis showed that *NEDD1* was significantly correlated with a common m6A modifiers writer, METTL3 (Figure 4C).

**Figure 4:** METTL3 regulates *NEDD1* through m6A modification. (A) Detection of *NEDD1* m6A methylation levels in DLBCL and nonneoplastic tissues by MeRIP‐qPCR. (B) Detection of *NEDD1* m6A methylation levels in AHH‐1, SU‐DHL‐8, and OCI‐LY1 cells. (C) Pearson's correlation analysis of *METTL3* and *NEDD1* in DLBCL cells analyzed in GEPIA. (D) The mRNA expression of *METTL3* and *NEDD1* in AHH‐1, SU‐DHL‐8, and OCI‐LY1 cells by RT‐qPCR. (E) The mRNA and protein expression of METTL3 and NEDD1 in DLBCL cells in response to si‐NC, si‐METTL3, si‐METTL3 + NC‐OE, and si‐METTL3 + NEDD1‐OE by RT‐qPCR and western blot. (F) Detection of *NEDD1* m6A methylation levels in SU‐DHL‐8 and OCI‐LY1 cells in response to si‐NC or si‐METTL3 by MeRIP‐qPCR. (G) Pearson's correlation of analysis *YTHDF1* and *NEDD1* in DLBCL cells analyzed in GEPIA. (H) The effectiveness of *YTHDF1* silencing in DLBCL cells using RT‐qPCR. (I) The protein expression of NEDD1 in DLBCL cells in response to silencing of YTHDF1 using western blot. (J) Stability of *NEDD1* mRNA in DLBCL cells infected with si‐YTHDF1. Mean ± SD (paired *t*‐test, one‐way or two‐way ANOVA). *p < .05 versus nonneoplastic tissues, AHH‐1 cells, or si‐NC group; #*p* < .05 versus si‐METTL3 + NC‐OE. DLBCL, diffuse large B‐cell lymphoma; m6A, N6‐methyladenosine; RT‐qPCR, quantitative real‐time polymerase chain reaction; SD, standard deviation.

RETRACTED

To investigate whether METTL3 partook in the pathogenesis of DLBCL by regulating *NEDD1* m6A methylation, the *METTL3* and *NEDD1* expression in DLBCL and AHH‐1 cells were measured using RT‐qPCR. *METTL3* and *NEDD1* were found to be overexpressed in both DLBCL cells relative to AHH‐1 cells (Figure 4D). DLBCL cells were then infected using si‐NC, si‐METTL3, si‐METTL3 + NC‐OE, or si‐METTL3 + NEDD1‐OE and validated for transfection efficiency. RT‐qPCR and western blot assays demonstrated that silencing of METTL3 downregulated the expression of METTL3 and NEDD1 in SU‐DHL‐8 and OCI‐LY1 cells, whereas NEDD1‐OE enhanced the expression of NEDD1 in the presence of si‐METTL3 (Figure 4E). MeRIP qPCR assay showed that depletion of METTL3 decreased the level of m6A methylation in *NEDD1* mRNA (Figure 4F). It was thus presumed that silencing of METTL3 in SU‐DHL‐8 and OCI‐LY1 cells downregulated *NEDD1* expression via m6A modification.

Pearson's correlation analysis in GEPIA revealed that *YTHDF1*, an m6A reader, had a high correlation with *NEDD1* in DLBCL (Figure 4G). The DLBCL cells were then infected with si‐YTHDF1, and the efficiency was verified using RT‐qPCR (Figure 4H). Reduced protein expression of NEDD1 was found in SU‐DHL‐8 and OCI‐LY1 cells with YTHDF1 knockdown (Figure 4I). To determine whether YTHDF1 governed the mRNA stability of *NEDD1* in cells, we performed RNA stability analysis. The half‐life of *NEDD1* was shortened in SU‐DHL‐8 and OCI‐LY1 cells in response to YTHDF1 knockdown (Figure 4J).

### 3.5 NEDD1 abolishes the repressive effects of si‐METTL3 on DLBCL cell aggressiveness

The results of EdU assays presented that depletion of METTL3 inhibited the proliferation of SU‐DHL‐8 and OCI‐LY1 cells and that NEDD1 overexpression mitigated the repressive effect of si‐METTL3 on cell proliferation (Figure 5A). Silencing of METTL3 weakened the mobility of DLBCL cells, whereas ectopic expression of NEDD1 reversed the effect of si‐METTL3 to elevate cell migration and invasion (Figure 5B,C). The apoptosis rate of SU‐DHL‐8 and OCI‐LY1 was induced by knockdown of METTL3, while NEDD1 ectopic expression mitigated the proapoptotic effect of METTL3 silencing on SU‐DHL‐8 and OCI‐LY1 cells (Figure 5D).

RETRACTED

**Figure 5:** Ectopic expression of NEDD1 reverses the repressive effects of METTL3 loss on DLBCL cell proliferation. (A) DLBCL cell proliferation examined using EdU assay. (B) DLBCL cell migration was measured using Transwell migration assay. (C) DLBCL cell invasion measured using Transwell invasion assay. (D) DLBCL cell apoptosis was measured using flow cytometry. Mean ± SD (two‐way ANOVA). *p < .05 versus si‐NC group, #*p* < .05 versus si‐METTL3 + NC‐OE group. ANOVA, analysis of variance; DLBCL, diffuse large B‐cell lymphoma; EdU, 5‐ethynyl‐2′‐deoxyuridine; SD, standard deviation.

### 3.6 *NEDD1* promotes DLBCL tumor growth and immune evasion in vivo

The impact of METTL3 and NEDD1 on DLBCL tumorigenesis was examined in vivo (only SU‐DHL‐8 cells were used for in vivo experiments to reduce unnecessary sacrifices). Silencing of METTL3 significantly reduced tumor weight, while NEDD1‐OE elevated tumor weight (Figure 6A,B). The expression of ki‐67 was examined in tumor tissues, and it was observed that depletion of METTL3 resulted in the inhibition of the proliferative activity of tumor tissues, whereas ectopic expression of NEDD1 reversed the impact of silencing of METTL3 to increase the growth of tumors (Figure 6C). Finally, the expression of TGF‐β and IL‐10 immunosuppressive factors were detected in tumor tissues. Si‐METTL3 inhibited the levels of TGF‐β and IL‐10, while si‐METTL3 + NEDD1‐OE increased their release in tumor tissues (Figure 6D,E), indicating that METTL3 promoted immune escape in DLBCL by upregulating *NEDD1*.

**Figure 6:** Ectopic expression of NEDD1 reverses the repressive effects of METTL3 loss on tumor growth in vivo. (A) Representative tumor images. (B) The tumor weight. (C) Immunohistochemical detection of proliferative activity in tumor tissues. (D) The protein expression of TGF‐β and IL‐10 in tumor tissues examined using western blot. (E) The levels of TGF‐β and IL‐10 in mouse tumor tissues using ELISA. Mean ± SD (one‐way or two‐way ANOVA). *p < .05 versus si‐NC group, #*p* < .05 versus si‐METTL3 + NC‐OE group. ANOVA, analysis of variance; DLBCL, diffuse large B‐cell lymphoma; ELISA, enzyme‐linked immunosorbent assay; IL, interleukin; SD, standard deviation; TGF‐transforming growth factor.

RETRACTED

## 4 DISCUSSION

Over the past decade, outstanding progress has been achieved in the understanding of the DLBCL pathogenesis, and the alterations involve epigenetic remodeling, block of differentiation, as well as immune escape.^17^ However, the molecular mechanism through which several elements of tumor microenvironment conferring aggressiveness remains poorly understood.^18^ We revealed here that NEDD1 was promoted in DLBCL tissues and cells. We then conducted functional experiments to examine the involvement of NEDD1 in DLBCL. NEDD1 was revealed to be an oncogene in DLBCL, and its depletion contributed to decreased cell proliferation and mobility, and enhanced T cell function via the impairment of the Hedgehog pathway. NEDD1 was found to be regulated by the m6A writer METTL3 and the reader YTHDF1 in DLBCL. Lastly, the in vitro findings were substantiated in vivo: the injection of DLBCL cells with METTL3 knockdown resulted in smaller tumors in mice, which was reversed by NEDD1 overexpression.

Fujita et al.^19^ have reported that intraperitoneal delivery of a siRNA targeting NEDD1 prolonged the survival of scirrhous gastric cancer model mice. Here, by using siRNA targeting NEDD1, we found that the viability, migration, and invasion of DLBCL were remarkably reduced, whereas the apoptosis rate was significantly restored. Hedgehog signaling proteins have been documented to commonly expressed in DLBCL.^20^, ^21^ Intriguingly, Cascio et al. found that in patient samples, cancer‐associated mesenchymal stem cells inversely correlated with the presence of intratumoral CD8^+^ T cells, while the Hedgehog inhibitor therapy reduced myeloid cell presence and expression of TGF‐β and restored the response to immune checkpoint inhibitor therapy.^22^ The regulatory mechanism of NEDD1 on the Hedgehog signaling was then validated in the present study. Here, we also found that depletion of NEDD1 successfully lowered the levels of TGF‐β and IL‐10 in DLBCL cells and elevated the killing effects of T cells on the DLBCL cells. We believed that the effects of si‐NEDD1 on DLBCL cells were elicited through the disruption of the Hedgehog signaling.

In addition to the downstream mechanism of NEDD1, we deciphered the upstream mechanism leading to NEDD1 overexpression in DLBCL as well. Our MeRIP‐qPCR analyses substantiated the m6A modification of *NEDD1* in DLBCL tissues and cells, which indicated that the dysregulation of NEDD1 was related to the m6A modification. METTL3 was revealed as a potential oncogene for hematologic system tumors.^23^ We observed here the positive correlation between *NEDD1* and *METTL3* in the bioinformatics website. Moreover, loss of METTL3 using a siRNA contributed to the downregulation of *NEDD1* mRNA expression and m6A modification level in DLBCL cells. YTHDF1 is the most versatile and powerful reader protein of m6A‐modified RNA and manipulates the expression of its targets by encouraging translation or modulating the stability of mRNA, thereby involving in tumor biology and nontumor lesions.^24^ Here, we also found that YTHDF1 downregulation repressed the *NEDD1* mRNA stability. Consistently, overexpression of METTL3 induced cell proliferation in vitro and enhanced tumorigenicity in vivo by accelerating the translation of *CDC25B* mRNA through YTHDF1‐dependent m6A modification in cervical cancer as well.^25^

RETRACTED

In leukemia cell lines, METTL3 enhanced cell proliferation and cell cycle, and the knockdown of METTL3 induced apoptosis and differentiation of acute myeloid leukemia cells.^26^ Also, METTL3 modulated the secretion of TGF‐β1, thus suppressing TGF‐β‐induced epithelial‐mesenchymal transition.^27^ As the first discovered methyltransferase, METTL3 has been documented to methylate its target transcripts and participate in various physiological processes, including T cell homeostasis.^28^ Additionally, METTL3‐driven m6A modification of RNA promoted immunosuppression of tumor‐infiltrating myeloid cells.^29^ METTL3 mediated the m6A modification of hsa_circ_0079587 and promoted its circularization, while hsa_circ_0079587 attenuated CD8^+^ T cell‐mediated antitumor immunity in non‐small‐cell lung carcinoma, as evidenced by the compromised secretion of IFN‐γ and TNF‐α.^30^ Nevertheless, the mechanism of METTL3 on the T cell function has not been clearly established. It is notable from our rescue experiments that the tumor inhibiting effects of si‐METTL3 on DLBCL cells were reversed by NEDD1 in vitro and in vivo, further supporting that METTL3 is an upstream m6A modifier of NEDD1.

## 5 CONCLUSION

Our study collectively revealed that NEDD1 expedited DLBCL cell proliferation and invasion in vitro, and tumor growth in vivo. From the perspective of mechanism, we elucidated that METTL3 coordinated with YTHDF1 to regulate NEDD1 m6A modification in DLBCL cells to activate the Hedgehog signaling, leading to the immune evasion of DLBCL cells. These observations further suggested that NEDD1 might serve an attractive target for immunotherapy in DLBCL.

## AUTHOR CONTRIBUTIONS

**Lili Feng**: Conceptualization; data curation; project administration; software; writing—original draft. **Qinying Yan**: Data curation; formal analysis; methodology; supervision; writing—review & editing. **Hui Pan**: Data curation; investigation; software; validation; writing—review & editing. **Wodong Shi**: Formal analysis; methodology; supervision; visualization; writing—original draft.

RETRACTED

## CONFLICT OF INTEREST STATEMENT

The authors declare no conflict of interest.

## Data Availability

Data are available on request due to privacy/ethical restrictions.
